This article has been retracted.

# Analysis of Risk Factors and Nursing Intervention Measures Affecting Nutritional Status of Children with Crohn's Disease

**DOI:** 10.1155/2021/5416487

**Published:** 2021-10-11

**Authors:** Chao Fan, Jieyu You, Hongmei Zhao, Meizheng Zhan, Cui Gao, Hong Ye, Lichun Yi

**Affiliations:** Department of Gastroenterology and Nutrition, Hunan Children's Hospital, No. 86, Ziyuan Road, Yuhua District, Changsha, Hunan 410000, China

## Abstract

In recent years, the incidence of Crohn's disease (CD) in the Asia-Pacific region is gradually increasing, and the onset age is decreased at the same time. The relapse of illness and long course of disease easily lead to malnutrition, which will affect the treatment effect of the disease and even worsen the disease. Therefore, it is very important to find the risk factors affecting the nutritional status of children with CD and to carry out effective nursing intervention accordingly. In our study, a total of 180 children with CD who were admitted to our hospital from April 2017 to April 2020 were analyzed retrospectively. The multivariate analysis showed that Pediatric Crohn's Disease Activity Index (PCDAI), platelet (PLT), hemoglobin (HB), hematocrit (HCT), and albumin (ALB) were independent risk factors affecting the nutritional status of children with CD. The results of AUC showed that combined monitoring of the PCDAI score and the expression of PLT, HB, HCT, and ALB indexes was of great value to evaluate the nutritional status of children with CD. Finally, a series of nursing intervention measures were proposed based on these results. It provides a theoretical basis for improving the nutritional status of children with CD and promoting the clinical outcome.

## 1. Introduction

Crohn's disease (CD) is a chronic, recurrent, inflammatory disease occurring in the digestive system of unknown cause [1, 2]. It can involve the entire gastrointestinal tract from the mouth to the anus and is usually segmental and skipping in distribution. The lesion sites of children with CD are mostly distributed in the ileocolon and upper digestive tract, with the clinical manifestations of chronic diarrhea and abdominal pain [3, 4]. In addition, long-term inflammation of the gastrointestinal tract can also cause complications such as fistulas, abscesses, intestinal stenosis, obstruction, and perforation [5]. The disease can occur repeatedly and is hard to be cured, which seriously affects the growth and development of children.

Relevant statistics showed that more than 25% of CD patients were malnourished, which was influenced by insufficient nutrient intake, absorption disorders, intestinal dysfunction, and increased consumption of body [6, 7]. The earliest manifestation of malnutrition is the recent lack of weight gain or decline, and the severe manifestations are anemia and hypoproteinemia, which can lead to the deterioration of the general condition and the decline of the quality of life in children with CD [8]. Nutritional status is closely related to the degree of disease development. However, there are few reports on the nutrition of children's CD [9]. Therefore, the in-depth study of the risk factors affecting the nutritional status of children with CD and reasonable nutritional nursing intervention is essential in the clinical treatment and rehabilitation of children with CD. This study analyzed the risk factors affecting the nutritional status of children with CD and proposed relevant nursing interventions, which are reported as follows.

## 2. Materials and Methods

### 2.1. General Information

A total of 180 children with CD who were admitted to our hospital from April 2017 to April 2020 were analyzed retrospectively. There were 96 males and 84 females with an average age of (8.74 ± 2.33) years old.

### 2.2. Inclusion Criteria

The inclusion criteria are as follows: the diagnostic criteria of CD were based on the consensus opinion on diagnostic norms of inflammatory bowel disease in Children proposed by the Pediatric Inflammatory Bowel Disease Collaborative Group of Gastroenterology Group of Pediatric Society of Chinese Medical Association in 2010, age 7–12 years, and all parents were informed of the study and signed informed consent forms.

### 2.3. Exclusion Criteria

The exclusion criteria are as follows: the height and weight cannot be measured due to the disease itself and other reasons, children with comorbid other infectious diseases or systemic infections, children with other chronic conditions such as combined primary immunodeficiency disease, and children who had been transfused with plasma or human serum protein preparations within 4 weeks.

### 2.4. Methods

#### 2.4.1. Collect the Baseline Information

Through the electronic medical record, the specific conditions of the children were recorded, including age, gender, BMI, lesion location, lesion type, the presence or absence of perianal lesions, and the presence or absence of the intestinal surgery history. The lesion sites include the terminal ileum (L1), colon (L2), ileocolon (L3), ileum + upper digestive tract (L1 + L4), colon + upper digestive tract (L2 + L4), and ileocolon + upper digestive tract (L3 + L4). The lesion type included nonstenosis or nonpenetrating (B1), stenosis (B2), penetrating (B3), and stenosis + penetrating (B2 + B3).

#### 2.4.2. Evaluate the Recent Disease Severity in Children with CD

The Pediatric Crohn's Disease Activity Index (PCDAI) scale was used, which consists of six main items based on subjective symptoms, extraintestinal manifestations, abdominal examination, perianal lesions, weight and height, and laboratory tests. The above six dimensions were observed and scored for one week, and the sum of the 6 scores was calculated as the total score by multiplying the specified weights.

A PCDAI score of ≥10 was defined as clinical activity, a PCDAI score of 10–29 was defined as mild activity, 30–40 was defined as moderate activity, and 41–100 was defined as severe activity.

#### 2.4.3. Collect the Clinical Biochemical Indexes

Within 48 hours after admission, 5 ml peripheral venous blood of children with CD was collected within 48 hours after admission and collected in vacuum collection vessels containing anticoagulant (K2-EDTA) produced by BD Company in the United States. After full mixing, the levels of white blood cell (WBC), platelet (PLT), hemoglobin (HB), hematopoietic volume (HCT), and albumin (ALB) were detected by the Japanese SYS-MEXXS-1000I automatic hematology analyzer within 1 h.

### 2.5. The Diagnostic Criteria for Malnutrition

The screening tool for risk of nutrition in growth kids (STRONGkids) was used to evaluate four components, including subjective clinical evaluation, intake and loss of nutrition, high-risk disease, and loss of weight or difficulty in weight gain. The scores of each component were summed and ≤3 was considered as low nutritional risk and ≥4 as high nutritional risk.

### 2.6. Statistical Methods

All data were processed with SPSS 22.0 statistical software, and GraphPad prism 8 was used to make statistical graphs. Measurement data are expressed as mean ± standard deviation ($\bar{x}$ ± *s*), the independent sample *t*-test is used for comparison between groups, count data are expressed as (*n* (%)), and the chi-square (*χ*^2^) test is performed. Factors significant in univariate analysis were subjected to multiple logistic regression model analysis. The receiver operating characteristic (ROC) curve was drawn to study the predictive value of independent risk factors on children's nutritional risk and calculate the area under curve (AUC). The difference is statistically significant when *P* < 0.05.

## 3. Results

### 3.1. Baseline Data

Among the 180 subjects, 2 cases were older than 18 years old and 3 cases had incomplete general data. After elimination, 175 cases were finally included. The nutritional status of 175 children with CD was evaluated, and the average NRS2002 score was (3.21 ± 1.37). Among them, 106 cases were ≥3, accounting for 60.57%; 69 cases were less than 3 points, accounting for 39.43%. All patients were divided into high nutritional risk and low nutritional risk according to the NRS2002 score. The clinical characteristics of all patients are given in Table 1.

### 3.2. Univariate Analysis of Nutritional Status of Children with CD

Univariate analysis showed that there was no significant difference in age, gender, disease behavior, perianal lesions, history of intestinal surgery, and WBC between the high nutritional risk and the low nutritional risk (*P* > 0.05). BMI, lesion type, PCDAI, PLT, HB, HCT, and ALB of the high nutritional risk and the low nutritional risk were statistically significant (*P* < 0.05, Table 2).

### 3.3. Variable Assignment

The existence of nutritional risk was taken as the dependent variable, and the factors with significant differences in Table 2 were taken as independent variables into the logistic regression model. The assignments of the dependent variables and independent variables are given in Table 3.

### 3.4. Multivariate Analysis of the Nutritional Status of Children with CD

Multivariate analysis showed that PCDAI, PLT, HB, HCT, and ALB were the independent risk factors affecting the nutritional status of children with CD (*P* < 0.05, Table 4).

### 3.5. ROC Curve Analysis of the Changes in PCDAI, PLT, HB, HCT, and ALB Levels to Predict the Nutritional Risk of Children with CD

The ROC curve was used to analyze the value of changes in PCDAI, PLT, HB, HCT, and ALB levels in predicting the nutritional risk of children with CD. The AUC in the ROC curve of changes in PCDAI, PLT, HB, HCT, and ALB individually and jointly predicts that the nutritional risk of children with CD was 0.640/0.700/0.891/0.819/0.960 and 0.994. The AUC of each index is maximum by joint detection (*P* < 0.05, Table 5 and Figure 1).

## 4. Discussion

CD is a common inflammatory bowel disease, and the main pathological type is transmural inflammation [10]. As the intestinal tract is the main organ for nutrient absorption, there are significant nutritional risks and growth retardation in children with CD. The number of CD patients in children is increasing year by year. Compared with CD in adults, childhood CDs have a wider range of intestinal involvement and more invasive inflammation [11, 12]. Therefore, it is necessary to timely detect the children at risk of malnutrition and carry out early nutritional intervention to improve the prognosis of the disease and reduce the risk of clinical poor prognosis.

### 4.1. Analysis of Risk Factors Affecting the Nutritional Status of Children with CD

Nutritional risk refers to the risk that the existing or potential nutritional status affects the clinical outcome of diseases, which is closely related to the clinical outcome. In our study, the NRS2002 method was used to evaluate the nutritional status of 175 children with CD, and the results showed 60.57% children with score ≥3, which was higher than the incidence of nutritional risk of inpatients in previous studies (35.5%). This result indicated that children with CD generally had nutritional risk.

Furthermore, the possible risk factors were analyzed by the logistics regression model, and the results showed that the nutritional risk of children with CD was related to the change of the PCDAI score. Children were divided into the clinical remission stage, mild active stage, moderate active stage, and severe active stage by PCDAI [13]. During the active period, the loss of intestinal nutrients increased, and patients need to limit food intake in order to intestinal symptoms, so the incidence of nutritional risk was higher. The degree of inflammation in the active lesions increased significantly [14]. At this time, the more serious the damage of intestinal mucosa at the lesion, the smaller the area of intestinal mucosa digesting and absorbing nutrients, which result in nutrient absorption disorder [15]. The active inflammation will also cause protein loss, which will further reduce the concentration of serum albumin, thus increasing nutritional risk. The levels of PLT, HB, HCT, and ALB were also independent risk factors affecting the nutritional status of children with CD [16]. The count changes of serological PLT, HB, HCT, and ALB count have been proved to be used as nutritional evaluation indexes in clinic. Wu et al. found that the combination of Hb, Hct, and Alb with the clinical scale is helpful to judge the nutritional status of patients with pulmonary tuberculosis complicated with intestinal tuberculosis and can provide follow-up treatment [17].

### 4.2. Analysis of the Clinical Value of Risk Factors Affecting the Nutritional Status of Children with CD

In order to confirm the role of changes in the levels of PCDAI, PLT, HB, HCT, and ALB in the nutritional status of children with CD, we used the ROC curve to compare and analyze the value of individual and combined detection of various indexes in predicting the nutritional risk of children with CD. The results showed that the AUC of each index was the largest, and the combined monitoring of PCDAI score and the expression of four indexes was of a great value to evaluate the nutritional status of children with CD. However, due to the immature immune system and digestive system of newborns and the influence of age, there are great differences in individual manifestations of infection and inflammation [18]. So, there were some children's detection indicators even in the normal range, which may cover up the condition. Therefore, the evaluation of nutritional status by PCDAI, PLT, HB, HCT, and ALB still needs to combine the clinical manifestations, other laboratory indicators, and imaging examination results of children.

### 4.3. Nutritional Nursing Countermeasures for Children with CD

In the clinical work, nutritional intervention and nursing management of children with a high nutritional risk should be strengthened during the nursing process. First, establish a nutrition support group composed of doctors, nutritionists, nurses, and pharmacists. They should standardize application of various nutritional status assessment tools to comprehensively determine the energy metabolism, body composition, energy and protein balance, immune function, and muscle function of children.

Second, nurses need to carry out health education for children and their families according to the recommendations of dieticians and help their families to formulate standardized nutrition supply plans for children to ensure the effective supply of nutrients. Ask family members to give the child a high calorie, high quality protein, low fat, and easy to digest diet and avoid irritating, fried, milk, dairy products, and other foods. When supplementing nutrition, follow the principle of gradual, small meals. When necessary, various nutrients required by the body of the child need to be supplemented by enteral or parenteral routes.

Enteral nutrition is the preferred nutrition mode. But factor diet or total parenteral nutrition factor diet can be used as appropriate if enteral nutrition is insufficient or the children cannot tolerate it. Total parenteral nutrition should be given when the child has intestinal obstruction, gastric bleeding, or perforation. The supply time of EN and TPN: the time of nutritional support treatment should be determined according to the tolerance degree of different pipelines, the degree of disease development, and the state of consciousness of the children, which generally lasts 2–4 weeks. Nursing care of nutritional support therapy also includes many aspects. Too rapid infusion will lead to abnormal body temperature, vomiting, chest pain, and other discomforts in children. Therefore, it is necessary to infuse the nutrient solution evenly and in time and secure catheter properly. Parenteral nutrition requires regular pulse pressing flushing and strict aseptic operation principles [19].

In summary, PCDAI score, PLT, HB, HCT, and ALB levels are the independent risk factors for the nutritional status of children with CD. During the treatment period of children with CD, nutritional intervention and nursing management for children with high nutritional risk should be strengthened, in order to improve the nutritional status of children and accelerate clinical outcome. The deficiency of this study is that the sample size is small, and more sample sizes can be included in the future to further explore the specific molecular mechanism affecting the nutritional status of children with CD.

## Figures and Tables

**Figure 1:** ROC curve analysis of the changes in PCDAI, PLT, HB, HCT, and ALB levels to predict the nutritional risk of children with CD. The AUC in the ROC curve of changes in PCDAI, PLT, HB, HCT, and ALB individually and jointly predicting the nutritional risk of children with CD was 0.640/0.700/0.891/0.819/0.960 and 0.994. The AUC of each index is maximum by joint detection.

**Table 1:** Baseline information of 175 follow-up patients.

Clinical information		Number of cases	Proportion
Nutritional risk	High	106	60.57
	Low	69	39.43
Age	8.74 ± 2.33		
Gender	Male	94	53.71
	Female	81	46.29
BMI (kg/㎡)	20.33 ± 8.56		—
Lesion location	L1	39	22.29
	L2	36	20.57
	L3	84	48.00
	L1 + L4	7	4.00
	L2 + L4	5	2.86
	L3 + L4	4	2.29
Lesion type	B1	71	40.57
	B2	76	43.43
	B3	19	10.86
	B2 + B3	9	5.14
Perianal lesions	Yes	42	24.00
	No	133	76.00
PCDAI score	<10	79	45.14
	10–29	53	30.29
	30–40	36	20.57
	41–100	7	4.00
Intestinal surgery history	Yes	36	20.57
	No	139	79.43
WBC (×10^9^/L)	6.39 ± 3.15		—
PLT (×10^9^/L)	274.15 ± 96.37		—
HB (g/L)	118.33 ± 23.97		—
HCT (%)	35.17 ± 6.41		—
ALB (g/L)	37.58 ± 9.17		—

**Table 2:** Univariate analysis of nutritional status of children with CD.

Clinical information		High nutritional risk (*n* = 106)	Low nutritional risk (*n* = 69)	*χ* ^*2*^/*t*	*P*
Age		8.13 ± 1.98	8.52 ± 2.15	1.231	0.220
Gender	Male	56 (52.83)	38 (55.07)	0.085	0.771
	Female	50 (50.00)	31 (44.93)		
BMI (kg/㎡)		16.49 ± 4.37	19.98 ± 3.52	5.561	≤0.001
Lesion location	L1	28 (26.42)	11 (15.94)	17.463	0.004
	L2	14 (13.21)	22 (31.88)		
	L3	40 (37.74)	44 (63.77)		
	L1 + L4	6 (5.66)	1 (14.50)		
	L2 + L4	5 (4.72)	0 (0.00)		
	L3 + L4	3 (2.83)	1 (1.45)		
Lesion type	B1	40 (37.74)	31 (44.93)	2.417	0.490
	B2	46 (43.40)	30 (43.48)		
	B3	14 (13.21)	5 (7.25)		
	B2 + B3	6 (5.66)	3 (4.35)		
Perianal lesions	Yes	29 (27.36)	13 (18.84)	1.662	0.197
	No	77 (72.64)	56 (81.16)		
PCDAI score	<10	29 (27.36)	50 (72.46)	34.752	≤0.001
	10–29	41 (38.68)	12 (17.39)		
	30–40	30 (28.30)	6 (8.70)		
	41–100	6 (5.66)	1 (1.45)		
Intestinal surgery history	Yes	26 (24.53)	10 (14.49)	2.576	0.108
	No	80 (75.47)	59 (85.51)		
WBC (×10^9^/L)		6.13 ± 3.26	6.41 ± 3.11	0.565	0.573
PLT (×10^9^/L)		290.64 ± 56.26	251.19 ± 63.93	4.294	≤0.001
HB (g/L)		110.55 ± 16.87	124.35 ± 18.36	5.107	≤0.001
HCT (%)		31.58 ± 2.62	34.97 ± 4.52	6.275	≤0.001
ALB (g/L)		30.11 ± 2.74	36.08 ± 4.97	10.249	≤0.001

**Table 3:** Variable assignment for multivariate analysis of the nutritional status of children with CD.

Variable	The assignment
Dependent variable	
Nutritional risk	0 = low; 1 = high
Independent variables	
BMI	Input as actual BMI
Lesion location	*L*1 = 0, *L*2 = 1, *L*3 = 2, *L*1 + *L*4 = 3, *L*2 + *L*4 = 4, *L*3 + *L*4 = 5
PCDAI	<10 = 0, 10–29 = 1, 30–39 = 2, 40–100 = 3
PLT	Input as actual PLT
HB	Input as actual HB
HCT	Input as actual HCT
ALB	Input as actual ALB

**Table 4:** Multivariate analysis of the nutritional status of children with CD.

Factors	*β*	SE	Wald, *χ*^*2*^	*P*	OR	OR, 95% CI
BMI	−0.003	0.031	0.008	0.930	0.997	0.938–1.060
Lesion location	−1.270	0.981	7.758	0.129	0.881	0.090–1.876
PCDAI	−1.256	0.391	10.319	≤0.001	0.285	0.132–0.613
PLT	−0.013	0.002	29.558	≤0.001	0.987	0.983–0.992
HB	0.159	0.019	69.615	≤0.001	1.172	1.129–1.216
HCT	0.845	0.113	69.657	≤0.001	2.349	1.684–1.569
ALB	0.990	0.119	69.689	≤0.001	2.691	2.133–3.394

**Table 5:** Value of changes in PCDAI, PLT, Hb, HCT, and ALB levels in predicting nutritional risk in children with CD.

Predictor	Optimum threshold	Sensitivity	Sensitivity	AUC	95% CI
PCDAI	0.286	0.840	0.760	0.640	0.573–0.707
PLT	0.304	0.860	0.730	0.700	0.634–0.765
HB	0.173	0.880	0.700	0.891	0.850–0.931
HCT	0.461	0.840	0.740	0.819	0.756–0.883
ALB	0.196	0.870	0.760	0.960	0.940–0.979
Joint detection	0.297	0.980	0.790	0.994	0.988–0.999

## Data Availability

The data used to support the findings of this study are available from the corresponding author upon request.
